# The effects of the environmental protection tax law on heavily polluting firms in China

**DOI:** 10.1371/journal.pone.0261342

**Published:** 2021-12-16

**Authors:** Huwei Wen, Weifeng Deng, Quanen Guo

**Affiliations:** 1 Research Center of the Central China for Economic and Social Development, Nanchang University, Nanchang, Jiangxi, China; 2 Department of Economics, School of Economics and Management, Nanchang University, Nanchang, Jiangxi, China; 3 Department of Tourism Management, School of Tourism, Nanchang University, Nanchang, Jiangxi, China; China University of Mining and Technology, CHINA

## Abstract

In 2016, China implemented an environmental protection tax (EPTL2016) to promote the transformation and upgrading of heavily polluting industries through tax leverage. Using panel data of China’s listed companies, this study assesses the treatment effects of the EPTL2016 on the transformation and upgrading of heavily polluting firms by incorporating the intermediary role of the financial market. The empirical findings show that the EPTL2016 significantly reduced the innovation investment and productivity of heavily polluting firms but had no significant effect on fixed-asset investment. Additionally, EPTL2016 reduced the supply of bank loans to heavily polluting firms and increased the value of growth options for private enterprises and the efficiency of the supply of long-term loans to heavily polluting firms. Although the environmental policy of EPTL2016 benefits the transformation and upgrading of heavily polluting industries in many aspects, it generally hinders the industrial upgrading because of the reduction of bank loans.

## Introduction

China is under increasing pressure to conserve resources and protect the environment because of the size of its population and its rapidly growing economy [1]. Hence, to restrain the excessive consumption of environmental resources and meet its residents’ increasing environmental demands, China adopted various environment regulations to promote the transformation and upgrading of heavily polluting industries [2]. Tax policy targeting environmental protection, which is a market incentive instrument, is widely used to push micro-enterprises to invest in the environment and improve environmental performance [3]. In 2016, China promulgated its first law implementing an environmental protection tax to promote the development of an ecologically sustainable society, the “Environmental Protection Tax Law of the People’s Republic of China” (EPTL2016). This tax policy, which is legally binding on the environmental behavior of micro-enterprises, aims to internalize the costs of polluting emissions and develop a green economy in the long term.

The introduction of the EPTL2016 forces heavily polluting firms to pay a higher environmental tax for their pollution discharge. The environmental protection tax is more stringent than the pollutant discharge fee, and thus polluters cannot negotiate with local governments to reduce their payments [4]. Although the EPTL2016 presents an adverse shock, it may compel heavily polluting industries to upgrade their equipment and technology. On the one hand, polluters have a stronger incentive to invest in green technologies to comply with the environmental regulations, as in the Porter hypothesis [5]. On the other hand, the tax also affects the decisions and behaviors of enterprise stakeholders, especially commercial banks and capital market investors [6–8]. That is, heavily polluting firms may face severe financial constraints after policy intervention, leading to a lack of innovation capital for transformation and upgrading activities. Thus, we explore the following key questions: How does the EPTL2016 affect the transformation and upgrading of heavily polluting firms through financial markets? Does this policy affect the credit allocation of banks to enterprises and the equity value of heavily polluting firms?

The double-dividend effect of environmental taxes, first mentioned by the British welfare economist Pigou [9], refer to two effects. The first is the environmental dividend effect, by which the environmental tax can reduce environmental pollution [10]. The second is the social dividend effect, which consists of the efficiency dividend [11, 12], income distribution dividend [13, 14], and employment dividend [15–17]. The existing literature presents consistent conclusions on the environmental dividend effect of an environmental tax, though there is no consensus on the social dividend effect. Some studies hold opposing opinions that the environmental tax may introduce a redundant cost for firms [18], increase the unemployment rate [19], and lead to unequal income distribution [20].

Environmental regulation is the general term for the policies and measures formulated by the government to protect the environment [3]. We can divide the instruments of environmental regulation into three categories: command-and-control instruments, market incentive instruments, and voluntary environmental instruments [21]. The literature has two opposing viewpoints on the relationship between environmental regulation and enterprise competitiveness, specifically in the theory of compliance cost and the theory of innovation compensation. Neoclassical economists believe that environmental regulations can internalize the externality of pollution while increasing pollution costs, thereby reducing enterprise productivity and enterprise competitiveness. The theory of innovation compensation or the Porter hypothesis, holds that environmental regulations encourage firms to carry out innovation activities, apply green technologies, and improve their productivity.

Innovation activities, which require financial support, can realize the transformation and upgrading of heavily polluting firms [22]. However, obtaining funds for innovation through only internal financing channels is far from sufficient. The large, extensive financial market provides financial support for innovation activities and plays a vital role in the transformation and upgrading of enterprises. The bank credit market and the stock market represent the main debt financing and equity financing channels of listed enterprises, respectively [23]. In developing countries, capital markets are always imperfect, and enterprises depend more on the indirect financing of bank lending for long-term or risky investment activities [24]. Moreover, the financial market responds quickly to macroeconomic policies and is an important channel influencing the effect of environmental policy, or the EPTL2016 in this study.

Although a considerable body of literature investigates the effects of environmental taxes, further discussion on this topic remains necessary. First, prior studies focus mainly on macroeconomic effects such as the efficiency effect, employment effect, and distribution effects. However, these studies concentrate less on the effects on enterprise behavior, especially for heavily polluting firms. Environmental tax, as a micro-level policy, has a profound effect on firms’ investment and financing behaviors. Second, previous studies measure environmental tax mainly using alternative indicators such as emission charges or taxes related to the environment, which are highly subjective and endogenous. Third, most of the existing literature discusses the effect on enterprise behaviors while ignoring the role of the financial market. The EPTL2016 serves as a signal of enterprise operation pressure for heavily polluting firms, and the relevant stakeholders in the financial market respond quickly. Therefore, the financial market may affect the investment and financing behavior of heavily polluting firms.

Based on panel data of China’s listed companies, we investigate the effects of the EPTL2016 on the transformation and upgrading of heavily polluting firms by incorporating the intermediary role of the financial market. Specifically, we focus on the mechanism of bank loans, their allocation efficiency, and the equity value of enterprises. We treat the introduction of the EPTL2016 as a quasi-experiment and use the differences-in-differences (DID) method to assess the treatment effects of the EPTL2016 on the heavily polluting firms. The DID method can effectively avoid the endogeneity problem of the measurement of environmental taxes and identify causality. This study enriches the literature on environmental regulation theory and highlights bank credit and the equity value of enterprises to examine the heterogeneity of policy intervention effects for different enterprises. Our results provide an empirical basis for the reform of the environmental protection tax system. More importantly, this study contributes to the literature on the role of the financial market in the intervention effects of environmental policy.

## Environmental tax law and its effect on firm upgrading in theory

### Reform of environmental tax in China

China introduced several environmental protection laws, including the Environmental Protection Law, Radioactive Pollution Prevention Law, Environmental Impact Assessment Law, Clean Production Promotion Law, and so on. These laws cover almost all aspects of environmental pollution, but the environmental performance of heavily polluting firms has not improved enough to meet residents’ expectations. In the “Comprehensive Work Plan for Energy Conservation and Emission Reduction” issued by the State Council in May 2007, China first proposed to levy an environmental tax to correct the shortcomings of pollution charge fees and meet the goal of energy conservation and emission reduction. In 2014, the draft of the environmental protection tax law was submitted to the State Council, and public opinions were solicited from 2015 to 2016. In 2016, China’s first green tax law was passed and promulgated officially by the National People’s Congress.

An environmental protection tax, also known as a green tax, is a resource conservation and environmental protection policy. It is formulated based on the original system of pollution discharge fees and embodies the legislative principle of the tax shift. From this point of view, an environmental tax has a similar objective as the original pollutant discharge fee, mainly for air and water pollutants. Producers that discharge taxable pollutants pay an environmental protection tax. Compared with the pollution discharge fee, the environmental protection tax also increases the levy on excessive discharge from the centralized waste treatment site. The environmental protection tax expands the scope of taxable objects, strengthens control of pollutant emissions, and makes tax planning more specific and targeted. Overall, the environmental protection tax is a means of economic control over pollution.

### Theoretical effect of EPTL2016 on firm upgrading

The environmental policy may have an indirect effect on the decisions and behaviors of enterprise stakeholders. We argue that the promulgation of EPTL2016 serves as a signal for commercial banks and other financial institutions, which affect the financing and investment of heavily polluting firms. Bank loans are the most extensive external financing channel enterprises use [24]. We examine the effects of EPTL2016 on bank loans within heavily polluting industries. Heavily polluting firms face higher cleaning costs, which probably results in lower credit guarantees and higher default rates. Commercial banks are likely to reduce loans to heavily polluting firms after the EPTL2016, and banks must pay more attention to environmental and social risks in heavily polluting industries. Consequently, banks may reduce their lending quotas to heavily polluting firms. Hence, we propose the following hypothesis.

#### Hypothesis 1

The introduction of the EPTL2016 significantly reduces the bank credit of heavily polluting firms.

In a perfect capital market, capital flows mainly to more productive firms, and credit capital is no exception. Banks face challenges in allocating credit capital to efficient enterprises in heavily polluting industries because of asymmetric information. Thus, banks may choose to lend to companies with better financial performance. The EPTL2016 makes environment performance a strong constraint for enterprises, and the financial performance enterprises gain through pollution would be squeezed out. Thus, banks may refuse to lend to companies with high pollution and low productivity after the EPTL2016. In addition, commercial banks can obtain detailed environmental information about enterprises through other stakeholders after the policy, mitigating the information asymmetry between banks and enterprises. Hence, we propose the following hypothesis.

#### Hypothesis 2

The EPTL2016 has a positive effect on the efficiency of the supply of bank loans to heavily polluting industries.

Enterprises have the value of options in the face uncertainty, such as the growth and abandonment options [25]. According to the capital profit-seeking law and real options theory [26], investment is the main source of equity value. The timely expansion of fixed assets increases the value of the growth option when firms encounter better investment opportunities. When firms face poor investment opportunities, disposing of fixed assets increases the value of the abandonment option. Government policies have important external effects on the financing and investment activities of enterprises [23]. The EPTL2016 was a political signal that helped to reduce information asymmetry in investment activities. The promulgation of EPTL2016 placed pressure on heavily polluting firms to upgrade, which motivates executives to strengthen their self-discipline and exert more efforts in risky investment activities. Therefore, the EPTL2016 may enhance investment flexibility and investment efficiency through the information and competition effects. When faced with better investment opportunities, executives can quickly identify and grasp investment opportunities through information to execute growth options through the competition effect. Nevertheless, when facing poor investment opportunities, the information and competition effects cannot help enterprises reduce their investment quickly. Hence, we propose the following hypothesis.

#### Hypothesis 3

The EPTL2016 significantly increases the value of the growth options of heavily polluting firms but does not affect the value of the abandonment option.

Firm upgrading is a rather extensive and obscure concept. We define firm upgrading as the enterprise growth triggered by investment or innovation activities [27]. Although innovation is the fuse for firm upgrading, the increase in profits comes from the growth of the enterprise. Specifically, enterprises obtain above-average productivity through innovation investment and technology updating. The EPTL2016 could reduce the bank credit to heavily polluting industries, which may lead to a lack of funds for innovation and upgrading. Although the information and competition effects can improve the efficiency of credit allocation and increase equity value, we hold that the effects of credit supply reduction may be greater. Therefore, we propose the following hypothesis.

#### Hypothesis 4

The EPTL2016 has a negative effect on the upgrading of heavily polluting firms.

## Methodology and data

### Model specification

Following Wen and Lee [28], we adopt the DID method to assess the treatment effects of the EPTL2016 on bank loans and firm upgrading. Specifically, we divide enterprises into two groups and compare the group differences in the growth of firm upgrading before and after the policy. We can express the model as follows:

$$Y_{it}=\alpha_{i}+\beta_{1}Treat_{i}\times After_{t}+X_{it}\zeta +\lambda_{t}+\varepsilon_{it},$$ (1)

where *Y*_*it*_ is the dependent variable, which is firm upgrading and bank loans in our study. The variable *Treat*_*i*_ is the group dummy, which equals one if the firm belongs to a heavily polluting industry and zero otherwise. The variable *After*_*t*_ refers to the year dummy of policy intervention, and is equal to one after 2016 and zero otherwise. **X**_it_ represents several control variables that may affect the dependent variable. We are interested mainly in the regression-based DID estimator, *β*_1_, which is the treatment effect of the policy intervention.

We also employ a quasi-experiment design and investigate how the EPTL2016 affected the long-term loans of heavily polluting firms. Specifically, we use the following econometric model:

$$LongLoans_{it}=\alpha_{i}+\beta_{2}After_{t}\times FDummy_{it}+\beta_{3}FDummy_{it}+X_{it}\zeta +\lambda_{t}+\varepsilon_{it},$$ (2)

where *LongLoans*_*it*_ refers to the long-term loans of firm *i*. *FDummy*_*it*_ refers to the group dummy variables of the firms in heavily polluting industries, which we group using performance indicators. We focus on the coefficient of the interaction term, *β*_2_, which indicates the intervention effect of the EPTL2016 on the efficiency of the supply of long-term loans to heavily polluting industries.

Following Burgstahler and Dichev’s method [25], we use the following empirical econometric model to examine the effects of the EPTL2016 on the value of the growth options of heavily polluting firms:

$$\begin{array}{l} Ln(MV/BV)=\alpha_{0}+\alpha_{1}Gm+\alpha_{2}Gh+\alpha_{3}(E/BV)+\alpha_{4}Gm\times (E/BV)\\ \;+\alpha_{5}Gh\times (E/BV)+\alpha_{6}After+\alpha_{{}_{7}}After\times Gm+\alpha_{8}After\times Gh\\ \;+\alpha_{9}After\times (E/BV)+\alpha_{10}After\times Gm\times (E/BV)\\ \;+\alpha_{11}After\times Gh\times (E/BV)+Control^{'}{}_{it}\gamma +\sum Firm+\sum Year+\varepsilon_{it} \end{array}$$ (3)

where *MV* is the market value of the company’s equity. *BV* refers to net assets and *E* is the net profits of the firm. We divide the sample into three groups according to *E/BV*, which is the return on equity (*ROE*). *Gm* equals one if *E/BV* is in the middle group and zero otherwise. *Gh* equals one if *E/BV* is in the highest group and zero otherwise. When *Gh* equals one, the firm has high profitability. *Control*_*it*_ includes several control variables that may affect the equity value of enterprises. We test the coefficient of the interaction term (*After×(E/BV) ×Gh*). If *α*_11_ is significantly positive, then the EPTL2016 significantly increased the value of growth options of heavily polluting firms.

We employ the following model to study the effect of the EPTL2016 on the value of the abandonment option.


$$\begin{array}{l} Ln(MV/E)=\delta_{0}+\delta_{1}Dm+\delta_{2}Dh+\delta_{3}(BV/E)+\delta_{4}Dm\times (BV/E)\\ \;+\delta_{5}Dh\times (BV/E)+\delta_{6}After+\delta_{7}After\times Dm+\delta_{8}After\times Dh\\ \;+\delta_{9}After\times (BV/E)+\delta_{10}After\times Dm\times (BV/E)\\ \;+\delta_{11}After\times Dh\times (BV/E)+Control^{'}{}_{it}\gamma +\sum Firm+\sum Year+\varepsilon_{it} \end{array}$$ (4)

We divide the sample into three groups according to *BV/E*, which is the reciprocal of *ROE*. *Dm* equals one if *BV/E* is in the middle group and zero otherwise. *Dh* equals one if *BV/E* is in the highest group and zero otherwise. If *Dh* equals one, then the company’s profitability is poor. According to Hypothesis 3, the EPTL2016 environmental policy has no significant effect on the value of the abandonment option of firms with poor investment opportunities; hence, *δ*_11_ should be insignificant.

### Sample and data

We employ panel data of China’s A-share industrial listed firms, including 37 industries and a total of 2,786 enterprises. The heavily polluting industries as defined by the “Guidelines for Industry Classification of Listed Companies” (revised in 2012) and “Guidelines for the Disclosure of Listed Companies Environmental Information” (draft for comments) include coal mining and washing, oil and gas extraction, and so on. Our data set includes 996 heavily polluting firms in the treatment group and 1,820 other enterprises in the control group. We also investigate the effects of the EPTL2016 on the efficiency of the supply of long-term loans and the equity value of the 996 heavily polluting firms. Given that the EPTL2016 was introduced in 2016, we set the sample period from 2012 to 2019, which includes the four years before and after the policy intervention. We collected the financial data of firms from the Database of China Stock Market and Accounting Research. Some observations are lost during the regression analysis because of missing values.

We define firm upgrading as the enterprise growth triggered by investment or innovation activities. Although choosing the appropriate variables can be difficult, we employ *Innovation Input*, *Fixed-asset Investment*, and *Productivity* to reflect enterprise transformation and upgrading. *Innovation Input* is the natural logarithm of the firm’s R&D expense plus one, which is the best proxy variable that reflects the enterprise’s investment in upgrading. *Productivity* is the logarithm of the total factor productivity, which we measure following Levinsohn and Petrin’smethod [29]. It is a proxy variable that reflects the performance of the upgrading of the enterprise. We also use the variable *Fixed-asset Investment* to show the progress of enterprise upgrading, which we define as the cash payments for investing in fixed, intangible, and other long-term assets.

We also employ other dependent variables in the empirical analysis, including bank credit and equity value. Bank credit is the ratio of bank loans to total assets, which is the most important external financing source for enterprise upgrading. Equity value consists of the value of the growth options and the value of the abandonment option, all treated by logarithm. We add several control variables, as defined in Table 1. Table A1 in S1 File reports the descriptive statistics for the relevant variables. To eliminate the interference of extreme outliers on the empirical results, we winsorized some variables at the 1% level.

**Table 1:** Variable definition.

	Variables	Definition
Dependent variables	*Innovation Input*	Natural logarithm of the R&D expense plus one
	*Fixed-asset Investment*	Fixed-asset Investment/total assets
	*Productivity*	Natural logarithm of the total factor productivity
	*Bank credit*	100**×**Bank loans /total assets
	*Ln(MV/BV)*	Natural logarithm of the ratio of corporate equity value to net assets
	*Ln(MV/E)*	Natural logarithm of the ratio of corporate equity value to net profits
Independent variables	*lnAge*	Natural logarithm of the years that a firm has survived
	*lnSize*	Natural logarithm of the total assets
	*Education*	Proportion of undergraduates or above in total employees
	*Larst*	Percentage of shares owned by the largest shareholder
	*Cash*	Cash monetary assets /total assets
	*Lev*	Total debt/total assets
	*ROA*	Net income/total assets
	*State*	Equal one for state-owned enterprise and zero otherwise
	*Sep*	The difference between control and ownership of the listed company owned by the actual controller
	*Duality*	Equal one if the chairman and the general manager are not currently held by the same person and zero otherwise
	*KL*	Fixed assets/number of employees
	*Growth*	Growth rate of operating income

## Empirical results and analysis

### Effect of the EPTL2016 on bank credit

Table 2 shows the effects of the EPTL2016 on bank credit. Columns (1), (3), and (5) report the results of the regression-based DID estimation, while the other columns are the results for comparison. The coefficients of the control variables mostly meet the theoretical expectations or are not contradictory, thereby indicating that the empirical results are robust and relatively reliable. Although we can draw some interesting conclusions on the control variables, we focus on the treatment effects of the EPTL2016 or the coefficients of the interaction term.

**Table 2:** Effects of environmental protection tax law on bank credit.

Variables	*Long-term loan*		*Short-term loan*		*Total loans*	
	(1)	(2)	(3)	(4)	(5)	(6)
*Treat×After*	-0.497*	-0.867***	-0.544	-1.445***	-1.044**	-2.339***
	[-1.92]	[-3.80]	[-1.47]	[-4.35]	[-2.22]	[-5.58]
*lnAge*	2.504**	0.735	3.994**	-2.622***	6.725***	-1.869*
	[2.39]	[1.38]	[2.41]	[-3.29]	[3.21]	[-1.83]
*lnSize*	0.546***	0.439**	0.181	-0.054	0.746**	0.399
	[3.08]	[2.53]	[0.72]	[-0.22]	[2.37]	[1.29]
*Lev*	0.002	0.002	0.017**	0.019***	0.019**	0.022**
	[0.32]	[0.39]	[2.37]	[2.60]	[2.09]	[2.32]
*Growth*	-0.237***	-0.230***	-0.197***	-0.199***	-0.435***	-0.430***
	[-19.05]	[-18.63]	[-10.07]	[-10.26]	[-16.77]	[-16.66]
*Education*	-0.005	-0.006	0.004	0.002	0.0001	-0.003
	[-1.02]	[-1.11]	[0.54]	[0.27]	[-0.01]	[-0.27]
*Larst*	0.002	0.004	-0.017	-0.017	-0.014	-0.011
	[0.25]	[0.67]	[-1.53]	[-1.63]	[-0.99]	[-0.88]
*State*	-0.383	-0.315	-0.156	0.1	-0.44	-0.105
	[-0.94]	[-0.78]	[-0.26]	[0.17]	[-0.59]	[-0.14]
*Duality*	-0.305	-0.314	-0.442	-0.448	-0.808**	-0.822**
	[-1.49]	[-1.53]	[-1.42]	[-1.43]	[-2.14]	[-2.17]
*ROA*	0.0001	-0.001	-0.101***	-0.104***	-0.107***	-0.111***
	[-0.03]	[-0.04]	[-3.76]	[-3.90]	[-3.10]	[-3.23]
*Sep*	-0.024	-0.024	-0.032	-0.028	-0.059*	-0.054*
	[-1.53]	[-1.50]	[-1.23]	[-1.06]	[-1.84]	[-1.69]
*Constant*	-14.415***	-6.671**	-6.386	18.813***	-21.906**	11.809**
	[-3.00]	[-2.02]	[-0.89]	[3.93]	[-2.44]	[1.99]
Firm FE	Yes	Yes	Yes	Yes	Yes	Yes
Year FE	Yes	NO	Yes	No	Yes	No
N	15828	15828	15828	15828	15828	15828
Adj. R-sq	0.026	0.023	0.017	0.015	0.032	0.029

Notes: The numbers in bracket is T value. The asterisk represents the significance level

***(1%)

**(5%), and

*(10%).

The results show that the EPTL2016 significantly reduced bank loans to heavily polluting firms. When the dependent variables are the long-term or total loans, the coefficients of *Treat×After* are significantly negative, though they are insignificant in Column (3) for the dependent variable short-term loans. These results indicate that the EPTL2016 significantly reduced the long-term loans to heavily polluting firms, though the effect on short-term loans is unclear. Overall, the availability of bank loans for heavily polluting enterprises declined and these enterprises may suffer financing constraints. Long-term loans are the most important financing channel for innovation activities, so the EPTL2016 policy may hinder the innovation investment of these firms, thereby impeding industrial upgrading.

### Effects of the EPTL2016 on the allocation efficiency of long-term loans

We next use a sample of 996 firms in heavily polluting industries and investigate the effects of the EPTL2016 on the allocation efficiency of long-term loans. Specifically, we regress the variable long-term loans on the interaction terms between the time dummy variables (*After*) and group variables (*FDummy*). With this analysis, we aim to clarify the characteristics of the companies to which long-term credit prefers to flow. Table 3 summarizes the empirical results.

**Table 3:** Effects of EPTL2016 on the efficiency of the supply of long-term loans.

Variables	Dependent Variable: *long-term loan*					
	(1) TFP	(2) Innovation	(3) ROA	(4) Size	(5) State	(6) Political
*FDummy*	-0.715*	0.435	-0.384	4.831***		-0.229
	[-1.84]	[0.28]	[-0.79]	[13.03]		[-0.49]
*After×FDummy*	0.413	0.329	1.147**	-1.229***	-1.213***	0.79
	[0.86]	[0.59]	[2.51]	[-2.62]	[-2.60]	[1.27]
*lnAge*	5.642**	5.237**	4.957**	3.235	4.035*	5.402**
	[2.55]	[2.39]	[2.28]	[1.50]	[1.82]	[2.47]
*lnSize*	0.842***	0.830***	0.689**	0.487*	0.708**	0.831***
	[2.68]	[2.85]	[2.34]	[1.66]	[2.39]	[2.88]
*Lev*	0.0001	-0.005	-0.005	-0.007	-0.005	-0.005
	[-0.03]	[-0.75]	[-0.78]	[-1.14]	[-0.74]	[-0.76]
*Growth*	-0.249***	-0.252***	-0.253***	-0.083***	-0.251***	-0.252***
	[-12.32]	[-13.80]	[-13.73]	[-5.03]	[-13.70]	[-13.79]
*Education*	-0.006	-0.007	-0.008	-0.008	-0.007	-0.007
	[-0.91]	[-1.06]	[-1.10]	[-1.16]	[-1.06]	[-1.05]
*Larst*	0.002	0.006	0.005	0.007	0.01	0.007
	[0.15]	[0.49]	[0.40]	[0.57]	[0.73]	[0.51]
*State*	0.039	-0.374	-0.466	-0.632	0.281	-0.406
	[0.06]	[-0.60]	[-0.74]	[-1.08]	[0.42]	[-0.65]
*Duality*	-0.658*	-0.523	-0.532	-0.403	-0.508	-0.509
	[-1.68]	[-1.42]	[-1.44]	[-1.14]	[-1.38]	[-1.39]
*ROA*	0.001	-0.016	-0.027	-0.015	-0.01	-0.015
	[0.02]	[-0.50]	[-0.64]	[-0.49]	[-0.32]	[-0.49]
*Sep*	-0.012	-0.039	-0.04	-0.044	-0.029	-0.039
	[-0.40]	[-1.43]	[-1.45]	[-1.64]	[-1.07]	[-1.42]
Firm FE	Yes	Yes	Yes	Yes	Yes	Yes
Year FE	Yes	Yes	Yes	Yes	Yes	Yes
N	4550	5301	5301	5301	5301	5301
Adj. R-sq	0.032	0.034	0.035	0.099	0.035	0.034

Notes: The numbers in the bracket is the T value. The asterisk represents the significance level

***(1%)

**(5%), and

*(10%).

The variables of *TFP*, *Innovation*, *ROA*, *Size*, *Sate*, and *Political* are binary variables, which are equal to one for enterprises with high productivity, enterprises with continuous R&D investment, enterprises with a high return on assets, large-scale enterprises, state-owned enterprises, and politically connected enterprises, respectively.

The coefficients of the interaction terms in Columns (1) and (2) are positive but insignificant, and no evidence indicates that banks prefer productive and innovative firms after the EPTL2016. In Column (3), the coefficient of *After×FDummy* is significantly positive at the 5% level, indicating that the introduction of the EPTL2016 led to a preference for lending to profitable companies. Credit discrimination according to ownership type and size continues to exist in the lending market and led to some adverse effects on the availability of bank loans for investment activities [30–32]. In Columns (4) and (5), the coefficients of *After×FDummy* are significantly positive at the 1% level, which suggests that the EPTL2016 alleviated the phenomenon of scale and ownership discrimination in credit allocation. In addition, Column (6) shows that banks did not lend more to politically connected companies when the supply of bank loans was falling.

The above results indicate that the EPTL2016 reduced the supply of bank loans, but alleviated the phenomenon of credit discrimination and improved the efficiency of credit allocation to heavily polluting industries, which has two types of effects on firm upgrading. Although banks reduced the credit quota to heavily polluting firms, the improved allocation efficiency provides financing support for the long-term innovation investment of highly profitable enterprises, which may help firms upgrade their equipment and upgrade overall. In addition, smaller enterprises and private enterprises have better access to credit capital, which they can use to update fixed equipment and adopt cleaning technology, thus promoting firm upgrading. Under the EPTL2016 policy intervention, banks reduced their long-term loans to heavily polluting industries, while improving their allocation efficiency of bank credit, thus causing two opposing effects on firm upgrading.

### Effects of the EPTL2016 on equity value

We examine how the EPTL2016 policy affected the corporate valuations of stock market investors by employing the growth options and abandonment option value models. We also divide the sample into two subsamples according to firm ownership type. Columns (1) to (3) in Table 4 show the empirical results of the growth options value model, while the other columns report the results of the abandonment option value model.

**Table 4:** Effects of environmental protection tax law on the equity value.

Variables	Dependent Variable: *Ln (MV/BV)*			Variables	Dependent Variable: *Ln (MV/E)*		
	(1) Full	(2) SOEs	(3) Non-SOEs		(4) Full	(5) SOEs	(6) Non-SOEs
*Gh*	0.381***	0.235***	0.460***	*Dh*	0.321***	0.595***	0.148
	[9.87]	[4.29]	[9.27]		[4.94]	[7.46]	[1.56]
*Gm*	-0.073	-0.103	-0.019	*Dm*	-0.027	-0.157	0.006
	[-1.21]	[-1.11]	[-0.26]		[-0.38]	[-1.34]	[0.07]
*After*	-0.723***	-0.704***	-0.706***	*After*	-0.702***	-0.736**	-0.651***
	[-16.19]	[-9.44]	[-12.34]		[-4.56]	[-2.54]	[-4.23]
*E/BV*	-0.538***	-1.149***	-0.312***	*BV/E*	0.009***	0.009***	0.009***
	[-4.80]	[-5.52]	[-2.97]		[36.57]	[29.45]	[20.11]
*Gm×(E/BV)*	3.429***	4.132***	3.224***	*Dm×(BV/E)*	0.007	0.028***	-0.003
	[3.79]	[2.78]	[3.02]		[1.02]	[2.77]	[-0.31]
*Gh×(E/BV)*	0.099***	0.474***	0.092***	*Dh×(BV/E)*	0.000***	0.001***	0.000*
	[3.73]	[3.11]	[3.52]		[4.30]	[4.35]	[1.73]
*After×Gh*	-0.023	0.093*	-0.243***	*After×Dh*	-0.019	0.107	-0.078
	[-0.68]	[1.65]	[-4.40]		[-0.12]	[0.37]	[-0.54]
*After×Gm*	-0.003	0.098	-0.102	*After×Dm*	-0.068	0.105	-0.183
	[-0.04]	[0.88]	[-1.11]		[-0.41]	[0.36]	[-1.05]
*After×(E/BV)*	-0.148***	0.214	-0.172***	*After×(BV/E)*	0.011	0.037	-0.005
	[-3.73]	[1.23]	[-4.14]		[0.48]	[0.82]	[-0.23]
*After×(E/BV)×Gm*	-0.448	-2.135	0.357	*After×(BV/E)×Dm*	-0.009	-0.036	0.01
	[-0.42]	[-1.25]	[0.28]		[-0.39]	[-0.81]	[0.42]
*After×(E/BV)×Gh*	0.122**	-0.610***	1.115***	*After× (BV/E) ×Dh*	-0.011	-0.037	0.005
	[2.09]	[-2.74]	[4.24]		[-0.49]	[-0.82]	[0.23]
*Controls*	Yes	Yes	Yes	Controls	Yes	Yes	Yes
Firm /Year FE	Yes	Yes	Yes	Firm/Year FE	Yes	Yes	Yes
N	5237	1939	3298	N	4661	1690	2971
Adj. R-sq	0.5	0.493	0.565	Adj. R-sq	0.828	0.86	0.821

Notes: The numbers in the bracket is the T value. The asterisk represents the significance level

***(1%)

**(5%), and

*(10%).

For the growth options value model, the coefficients of *After×(E/BV)×Gh* are significantly positive at the 5% level for the full sample and the subsample of non-state-owned enterprises (non-SOEs), while the coefficient for SOEs is significantly negative at the 1% level. The results indicate that the value of growth options of non-SOEs improved through the information and competition effects. Conversely, the value of the growth options of SOEs decreased significantly, suggesting that the EPTL2016 did not improve the investment efficiency of SOEs. For the abandonment option value model, all the coefficients of *After×(BV/E) ×Dh* are insignificant, indicating that the policy did not cause an increase in the value of the abandonment option when firms face poor investment opportunities. Overall, Hypothesis 3 is established.

The different effects of the EPTL2016 on the value of growth options between SOEs and non-SOEs are not contradictory. When firms have better investment opportunities, market competition prompts the executives of non-SOEs to invest in projects with a positive net present value in a timely manner, thereby increasing the value of growth options. The weak management of SOEs leads to low investment efficiency and low investment flexibility, and the EPTL2016 cannot improve or even worsen the investment efficiency of SOEs through the information effect or competitive threat. Moreover, executives may choose to postpone some good investment opportunities, thereby reducing the value of growth options [33].

### Effects of the EPTL2016 on firm upgrading

The desired intervention effect of EPTL2016 is to facilitate innovation or technological updating of heavily polluting firms, which ultimately improves the productivity of such enterprises. However, the policy increased the financial constraints of heavily polluting enterprises, thereby leaving them without funds innovation investment and hindering long-term and risky investment activities. Hence, to examine whether the EPTL2016 policy hinders firm upgrading, we regress the proxy variables of firm upgrading on the interaction term between the group dummy (*Treat*) and the time dummy (*After*). We report the results in Table 5.

**Table 5:** Effect of environmental protection tax law on firm upgrading.

Variables	*Innovation Input*		*Productivity*		*Fixed-asset investment*	
	(1)	(2)	(3)	(4)	(5)	(6)
*Treat×After*	-0.560***	-0.384***	-0.159***	-0.133***	0.105	-0.077
	[-6.60]	[-4.92]	[-5.42]	[-4.77]	[0.55]	[-0.46]
*Lev*	0.005***	0.005***	0.009***	0.009***	-0.004	-0.001
	[3.62]	[3.51]	[12.60]	[12.61]	[-1.15]	[-0.31]
*lnAge*	-0.778	0.873***	0.11	0.124**	-4.532***	-6.955***
	[-1.58]	[4.50]	[0.90]	[2.25]	[-5.03]	[-17.17]
*ROA*	0.006	0.005	0.019***	0.019***	0.100***	0.097***
	[1.22]	[1.09]	[9.81]	[9.81]	[8.06]	[7.89]
*lnSize*	0.561***	0.616***	0.313***	0.318***	0.399***	0.306**
	[8.91]	[9.26]	[12.65]	[13.19]	[2.73]	[2.09]
*Education*	0.006***	0.006***	0.002***	0.002***	0.002	0.001
	[4.36]	[4.50]	[2.83]	[2.82]	[0.76]	[0.18]
*Larst*	-0.001	-0.002	-0.001	0.0001	0.018***	0.004
	[-0.58]	[-0.93]	[-1.33]	[-0.71]	[4.07]	[1.10]
*State*	-0.1	-0.163	-0.01	-0.003	-0.938***	-0.916***
	[-0.87]	[-1.44]	[-0.27]	[-0.08]	[-3.78]	[-3.72]
*Sep*	0.013**	0.012**	-0.003	-0.003	-0.014	-0.011
	[2.33]	[2.18]	[-1.61]	[-1.60]	[-1.37]	[-1.11]
*Cash*	0.002	0.003*	0.001	0.001	-0.038***	-0.034***
	[1.54]	[1.72]	[1.15]	[1.28]	[-7.79]	[-7.02]
*Duality*	0.01	0.008	-0.02	-0.02	0.329**	0.326**
	[0.15]	[0.13]	[-0.96]	[-0.97]	[2.29]	[2.26]
*Constant*	7.435***	1.223	0.564	0.407	9.022**	18.086***
	[4.45]	[0.93]	[0.88]	[0.90]	[2.33]	[6.46]
Firm FE	Yes	Yes	Yes	Yes	Yes	Yes
Year FE	Yes	No	Yes	No	Yes	No
N	15456	15456	14005	14005	15828	15828
Adj. R-sq	0.064	0.059	0.146	0.144	0.103	0.084

Notes: The numbers in the bracket is the T value. The asterisk represents the significance level

***(1%)

**(5%), and

*(10%).

The coefficients of *Treat×After* for innovation input and productivity are significantly negative at the 1% level, indicating that the EPTL2016 significantly reduced innovation investment and productivity. Firms in heavily polluting industries lack funds for innovation and risky investment activities after the adverse shock of the EPTL2016, resulting in a drop in innovation investment and productivity. That is, the introduction of the EPTL impeded the upgrading of heavily polluting firms. The regression coefficients of the interaction term (*Treat×After*) on fixed-asset investment are insignificant. The credit effect of the EPTL2016 may affect investment activities in two ways. Credit constraints prevent heavily polluting enterprises from blindly increasing their productive capital, thereby decreasing the investment rate and improving investment efficiency. In addition, credit constraints make it difficult for heavily polluting firms to upgrade to cleaner production facilities, thereby preventing such firms from upgrading to clean equipment and pollution-free production technologies. The insignificant effects of the EPTL2016 on fixed-asset investment indicate that two mechanisms may exist. Overall, although the EPTL2016 played an active role in limiting the expansion of inefficient capacity, achieving the goal of industrial upgrading in heavily polluting firms remains difficult.

## Further analysis and testing

### Heterogeneous analysis of firm size

Generally, small-scale enterprises face stronger financing constraints in the process of upgrading and are more sensitive to the effects of external financing channels. It is generally believed that small-scale enterprises have more difficulty surviving under the constraints of environmental regulations. However, the previous analysis revealed that the EPTL2016 reduced credit discrimination, thereby implying that the negative effect of the policy shock on the upgrading of small-scale enterprises is not larger than that of large-scale enterprises. Hence, we divide the sample into large-scale, medium-sized, and small-scale enterprises according to the quartile of the firm’s total assets. Then, we examine whether a significantly heterogeneous effect of the EPTL2016 on firm upgrading exists at different scales. Table 6 presents the results. All the coefficients of the interaction term *Treat×After* are significantly negative, thereby indicating that the EPTL2016 has significantly negative effects on the upgrading of different size enterprises. Moreover, we find no significant difference in the treatment effect for these three groups of firms. These results are consistent with the conclusion that the EPTL2016 reduced the scale discrimination of long-term loans.

**Table 6:** Heterogeneous effect of EPTL2016 on firm upgrading with different size.

Variables	*Innovation Input*			*Productivity*		
	(1) Large	(2) Medium	(3) Small	(4) Large	(5) Medium	(6) Small
*Treat×After*	-0.678***	-0.521***	-0.503***	-0.141**	-0.125**	-0.158***
	[-4.20]	[-3.49]	[-3.60]	[-2.49]	[-2.24]	[-2.83]
*Lev*	0.005	0.009***	0.003	0.009***	0.009***	0.009***
	[1.36]	[3.14]	[1.25]	[6.87]	[6.74]	[7.08]
*lnAge*	-0.225	-1.199	-0.9	0.288	0.235	-0.266
	[-0.38]	[-1.35]	[-1.55]	[1.48]	[1.37]	[-1.13]
*ROA*	0.006	-0.009	0.011	0.019***	0.020***	0.017***
	[0.70]	[-0.95]	[1.41]	[4.66]	[5.30]	[4.63]
*lnSize*	0.593***	0.537***	0.587***	0.275***	0.290***	0.352***
	[5.14]	[4.00]	[4.96]	[7.28]	[6.04]	[8.30]
*Education*	0.011***	0.0001	0.009***	0.002	0.002**	0.002
	[4.34]	[-0.01]	[3.88]	[1.49]	[2.03]	[1.54]
*Larst*	-0.005	-0.006	-0.001	-0.003*	-0.001	0.001
	[-1.31]	[-1.17]	[-0.27]	[-1.71]	[-1.05]	[0.60]
*State*	0.006	-0.036	0.098	-0.018	0.075	-0.002
	[0.04]	[-0.17]	[0.49]	[-0.26]	[1.11]	[-0.03]
*Sep*	0.011*	0.023**	0.012	0.001	0.002	-0.005*
	[1.74]	[2.28]	[0.86]	[0.33]	[0.67]	[-1.95]
*Cash*	0.004	0.003	0.001	0.002	0.001	0.0001
	[1.32]	[0.78]	[0.32]	[1.26]	[0.95]	[-0.32]
*Duality*	0.042	0.103	-0.019	-0.036	0.03	-0.017
	[0.33]	[0.91]	[-0.19]	[-0.84]	[0.75]	[-0.44]
*Constant*	4.844*	9.331***	7.193**	0.841	0.597	0.8
	[1.78]	[2.72]	[2.47]	[0.87]	[0.54]	[0.72]
Firm FE	Yes	Yes	Yes	Yes	Yes	Yes
Year FE	Yes	Yes	Yes	Yes	Yes	Yes
N	5144	5158	5154	4644	4691	4670
Adj. R-sq	0.071	0.055	0.084	0.15	0.14	0.157

Notes: The numbers in the bracket is the T value. The asterisk represents the significance level

***(1%)

**(5%), and

*(10%).

### Ownership type

Prior studies also show that upgrading activities are highly sensitive to changes in the external financing market, and it would be more difficult for private enterprises to operate under the constraints of environmental regulations. Hence, we divide the sample into three groups: state-owned, private, and foreign-owned enterprises. Then, we investigate whether the EPTL2016 has significantly heterogeneous effects based on ownership type.

The results in Table 7 show that all coefficients of the interaction terms are significantly negative, while the coefficient for private enterprises is no less than that of SOEs, indicating that the EPTL2016 hindered the upgrading of all heavily polluting firms, regardless of ownership. As the previous analysis shows, the EPTL2016 reduced ownership discrimination in long-term loans, and thus, the adverse effect of the EPTL2016 on private enterprises would not be greater than that of other enterprises. The results in Table 7 are also consistent with the conclusion that the policy increased the value of the growth options of private enterprises but reduced the value of growth options of SOEs.

**Table 7:** Heterogeneous effect of EPTL2016 on firm upgrading with different ownership.

Variables	*Innovation Input*			*Productivity*		
	(1) SOEs	(2) Private	(3) Foreign	(4) SOEs	(5) Private	(6) Foreign
*Treat×After*	-0.698***	-0.497***	-2.052**	-0.187***	-0.162***	-0.187*
	[-4.14]	[-4.96]	[-2.35]	[-4.07]	[-3.69]	[-1.96]
*Lev*	0.008***	0.003	0.013*	0.010***	0.008***	0.016***
	[2.64]	[1.42]	[1.86]	[8.46]	[8.26]	[2.83]
*lnAge*	-0.249	-0.477	-8.175*	0.37	-0.045	0.568
	[-0.14]	[-1.12]	[-1.68]	[1.00]	[-0.30]	[1.29]
*ROA*	0.023***	0.002	0.005	0.013***	0.027***	0.011
	[2.58]	[0.30]	[0.17]	[4.12]	[9.63]	[1.21]
*lnSize*	0.573***	0.575***	-0.086	0.293***	0.322***	0.037
	[3.72]	[7.88]	[-0.16]	[7.26]	[10.17]	[0.24]
*Education*	0.009***	0.004**	0.005	0.003***	0.001*	0.002
	[3.90]	[2.23]	[0.33]	[2.99]	[1.80]	[0.69]
*Larst*	0.002	0.007	-0.120**	-0.002	-0.002	-0.003
	[0.23]	[0.96]	[-2.21]	[-0.90]	[-0.73]	[-0.46]
*Sep*	0.012	0.009	0.07	0.001	-0.006*	-0.024**
	[0.88]	[1.14]	[1.35]	[0.39]	[-1.95]	[-2.14]
*Cash*	0.003	0.003	0.021	0.001	0.001	-0.001
	[0.66]	[1.32]	[1.63]	[0.32]	[1.36]	[-0.27]
*Duality*	0.119	-0.042	-0.299	0.017	-0.024	-0.013
	[0.79]	[-0.52]	[-1.00]	[0.34]	[-0.93]	[-0.14]
*Constant*	4.987	6.155***	47.559**	0.121	0.818	5.244
	[0.86]	[3.95]	[2.49]	[0.08]	[0.99]	[1.57]
Firm FE	Yes	Yes	Yes	Yes	Yes	Yes
Year FE	Yes	Yes	Yes	Yes	Yes	Yes
N	4440	8671	499	3779	8031	468
Adj. R-sq	0.049	0.075	0.197	0.112	0.163	0.168

Notes: The numbers in the bracket is the T value. The asterisk represents the significance level

***(1%)

**(5%), and

*(10%).

### Parallel trend test

An important prerequisite for unbiased DID estimation results is that the parallel trend hypothesis between the treatment and control groups is satisfied. In this study, the parallel trend means that there should be no systematic difference in the productivity of heavily polluting firms before and after the policy intervention. We therefore use the estimation coefficient of the dummy variables from 2013 to 2019 to investigate the dynamic effect on the productivity of heavily polluting enterprises. The specific test model is

$$\begin{array}{l} Productivity_{it}=\beta_{0}+\sum_{j=-3}^{3}\beta_{j}Treat_{i}\times year_{j}+\lambda X_{it}+\theta_{i}+\mu_{t}+\varepsilon_{it} \end{array}$$ (5)

Fig 1 shows the trend of the estimated value of the interaction term coefficient *β*_*j*_ in model 5, and presents the 95% confidence interval. The left half of the vertical dotted line is the difference in productivity between the treatment group and the control group before policy intervention, which indicates that the estimated *β*_*j*_ values in 2016 and previous periods are close to 0, including in the 95% confidence interval. That is, the estimated *β*_*j*_ values before the policy intervention are not significant. Thus, there was no significant change in the difference in productivity between the treatment and control groups in each period before the policy intervention, and the effect of the policy intervention generally meets the assumption of a parallel trend. After the policy intervention, the interaction term coefficient *β*_*j*_ is significantly negative, which indicates that the introduction of the EPTL2016 reduced the productivity of enterprises and hindered firm upgrading.

**Fig 1:** Parallel trend test of productivity of heavily polluting firms.

### Robustness test

Table 8 reports the results of the robustness test. Columns (1) to (3) are the DID regression results based on clustering standard errors. Column (1) to column (2) show the regression results of controlling firm and year fixed effects, and column (3) shows the regression results without controlling the year effect. The coefficients of the interaction item *Treat ×After* are all significantly negative at the 1% level, showing that the introduction of the EPTL2016 reduced the productivity of heavily polluting firms, and the result is robust.

**Table 8:** Robust test of the policy intervention on the productivity of heavily polluting firms.

Variables	Clustering standard error			Energy intensive firms as treatment group		
	(1)	(2)	(3)	(4)	(5)	(6)
*Treat×After*	-0.159***	-0.159***	-0.133***	-0.074***	-0.074**	-0.064**
	[-6.94]	[-6.13]	[-5.96]	[-4.18]	[-2.45]	[-2.19]
*lnAge*	0.11	0.11	0.124***	0.211***	0.211**	0.119**
	[1.63]	[1.28]	[3.05]	[2.91]	[2.06]	[2.25]
*Lev*	0.009***	0.009***	0.009***	0.008***	0.008***	0.008***
	[15.04]	[14.99]	[15.06]	[19.53]	[9.11]	[9.22]
*ROA*	0.019***	0.019***	0.019***	0.023***	0.023***	0.023***
	[10.97]	[9.30]	[10.97]	[18.59]	[12.20]	[12.17]
*lnSize*	0.313***	0.313***	0.318***	0.395***	0.395***	0.396***
	[18.22]	[13.45]	[19.43]	[34.35]	[16.93]	[17.40]
*Education*	0.002***	0.002***	0.002***	0.0001	0.0002	-0.001
	[3.07]	[3.13]	[3.09]	[-1.26]	[-0.75]	[-0.82]
*Larst*	-0.001*	-0.001	0.0001	-0.001**	-0.001*	0.0002
	[-1.68]	[-1.59]	[-0.83]	[-2.29]	[-1.91]	[-0.72]
*State*	-0.01	-0.01	-0.003	-0.008	-0.008	0.003
	[-0.34]	[-0.33]	[-0.11]	[-0.28]	[-0.23]	[0.08]
*Sep*	-0.003*	-0.003**	-0.003*	-0.001	-0.001	-0.001
	[-1.87]	[-2.04]	[-1.86]	[-1.29]	[-0.93]	[-0.89]
*Cash*	0.001	0.001	0.001	0.001**	0.001*	0.001*
	[1.50]	[1.63]	[1.63]	[2.18]	[1.67]	[1.77]
*Duality*	-0.02	-0.02	-0.02	-0.044***	-0.044**	-0.045**
	[-1.31]	[-1.19]	[-1.31]	[-3.05]	[-2.27]	[-2.31]
*_cons*	0.564	0.564	0.407	-1.487***	-1.487***	-1.242***
	[1.26]	[1.06]	[1.28]	[-4.71]	[-2.67]	[-2.95]
Year FE	Yes	Yes	No	Yes	Yes	No
Firm FE	Yes	Yes	Yes	Yes	Yes	Yes
N	14005	14005	14005	10989	10989	10989
Adj. R-sq	0.146	0.146	0.144	0.126	0.265	0.262

Notes: The numbers in the bracket is the T value. The asterisk represents the significance level

***(1%)

**(5%), and

*(10%).

The clustering standard errors in columns (1) to (3) are calculated at the level of industry, province and province respectively. Column (5) uses the robust standard errors.

In addition, we replace the treatment group sample by selecting six high-energy-intensive industries as the treatment group among the heavily polluting enterprises, and maintain the previous control group. Columns (4) to (6) are the DID regression results with the treatment groups of six energy-intensive industries. Columns (4) show the two-way fixed effect regression results and column (5) regress with robust standard error, and column (6) shows the regression results without controlling the year effect. The coefficients of the interaction terms all are significantly negative at the 5% level, which indicates that the introduction of the EPTL2016 significantly reduced the productivity of energy-intensive enterprises. That is, the previous conclusion is robust.

## Conclusions

The environmental pollution by heavily polluting industries seriously limited the sustainable development of China’s economy. Motivating heavily polluting firms to improve their environmental performance has been widely discussed by policy designers and scholars. Based on panel data of China’s A-share listed firms from 2012 to 2019, we apply the DID method to investigate the impact of the EPTL2016 on firm upgrading from the perspective of the intermediary role of the financial market.

The empirical evidence shows that although the EPTL2016 policy may help heavily polluting firms upgrade in many aspects, it also significantly reduced the innovation investment and productivity of heavily polluting firms. Under the policy intervention, banking institutions reduced the supply of loans to heavily polluting firms, which led to a decline in innovation investment and productivity. Admittedly, the policy may limit the blind expansion of production scale and encourage firms to upgrade their production equipment. We also find that the supply of long-term loans to heavily polluting industries is more efficient and the value of growth options for private firms increased after the EPTL2016 intervention. It provides financial support for the development of high-quality private firms because of the increase in the value of growth options. The heterogeneity analysis shows that the EPTL2016 reduced innovation investment and productivity for all heavily polluting enterprises, regardless of ownership and asset size. These results satisfy the parallel trend hypothesis, and the conclusions are robust based on a cluster standard error regression and an alternative treatment group.

The main finding in our study is that as banks tend to reduce the supply of loans to heavily polluting firms, these industries may be unable to obtain funds for innovation activities, thereby inhibiting their green upgrading and development in the long term. The findings of this study have some important implications. First, the formulation of the tax rate must adapt to the actual cost of the enterprise; that is, the tax cost must be greater than or equal to the income from the emission of pollutants, which will encourage firms to invest in green technology. Second, governments must design incentive policies that encourage heavily polluting firms to participate in innovation activities. The formulation of tax preference must fully consider the balance of interests between the environment and taxation, and reasonably adjust the scope of application of tax preferences, so tax can play a positive role in promoting environmental protection. Third, China should standardize and improve its green credit policy in case of blind expansion or lack of funds for innovation, and have a role in financial markets in allocating resources and avoid the excessive intervention of bank loans. Meanwhile, the government should guide the credit market and capital market to allocate capital more effectively, such that capital flows to efficient enterprises and promotes firm upgrading.

## Supporting information

S1 File (RAR)
